# CtBP2 is an independent prognostic marker that promotes GLI1 induced epithelial-mesenchymal transition in hepatocellular carcinoma

**DOI:** 10.18632/oncotarget.2915

**Published:** 2015-02-19

**Authors:** Xin Zheng, Tao Song, Changwei Dou, Yuli Jia, Qingguang Liu

**Affiliations:** ^1^ Department of Hepatobiliary Surgery, the First Affiliated Hospital of Xi'an Jiaotong University, Xi'an, Shaanxi 710061, China

**Keywords:** C-terminal binding protein 2, CtBP2, GLI family zinc finger 1, GLI1, Snail Family Zinc Finger 1, epithelial-mesenchymal transition, EMT, Hepatocellular carcinoma, HCC

## Abstract

C-terminal binding protein 2 (CtBP2) is a transcriptional co-repressor that promotes cancer cell migration and invasion by inhibiting multiple tumor suppressor genes that contribute to cell mobility and adhesion. In this investigation, we showed thatCtBP2 expression was increased significantly in HCC tissues when compared to matched normal adjacent liver tissues. We also showed that CtBP2 expression is associated with worse HCC patient prognosis after liver resection. CtBP2 over-expression induced epithelial-mesenchymal transition (EMT) in Huh7 cells and, correspondingly, silencing CtBP2 suppressed EMT in MHCC97H cells. ChIP assays revealed that GLI1 increased CtBP2 transcription by directly binding its promoter. Furthermore, interaction of CtBP2 and Snail Family Zinc Finger 1 (SNAI1), both of which were found to be positively regulated by GLI1, was confirmed by Co-IP assay. SNAI1 knockdown revealed that SNAI1 was essential for CtBP2 induction of the EMT phenotype of HCC cells, and CtBP2 knockdown reversed GLI1-SNAI1 driven EMT in Huh7 cells. Finally, *in vivo* experiments demonstrated that enhanced CtBP2expression promoted HCC xenograft growth and induced EMT. In conclusion, CtBP2 may serve as a prognostic marker for post liver resection HCC and may play a role during GLI1-driven EMT as a transcriptional co-repressor of SNAI1.

## INTRODUCTION

Hepatocellular carcinoma (HCC) is the most common primary liver cancer subtype [1] and one of the major causes of mortality in developing countries [2]. Current curative therapies, including liver resection and liver transplantation, have a high rate of post-surgical recurrence [3]. HCC recurrence occurs because of both primary tumor metastatic dissemination prior to surgery and new neoplasm development in the remaining liver tissues after surgery. Because of the high rate of recurrence, the postsurgical prognosis of HCC patients is extremely poor. Therefore, better understanding of the molecular mechanisms underlying HCC recurrence and metastasis and identification of biomarkers that can predict postsurgical HCC outcome is urgently needed.

C-terminal binding protein (CtBP) was first established as a phosphoprotein bound to the C terminal of the E1A protein [4]. The CtBP family consists of two genes, CtBP1 and CtBP2, which are conserved among both vertebrates and invertebrates [5]. CtBPs reportedly function primarily as transcriptional co-repressors and play important roles in development and tumorigenesis [6–9]. CtBPs have also been demonstrated to function as context-dependent transcriptional activators [10, 11]. A growing body of evidence indicates that CtBP2 is aberrantly upregulated in a variety of cancers and that its expression promotes cancer progression. Zhang *et al*. reported that CtBP2 was overexpressed in prostate cancer tissues and associated with poor outcome and several indicators of malignancy, including elevated serum PSA levels, advanced tumor stages and higher Gleason scores. Zhang *et al*. also reported that CtBP2 expression promoted prostate cancer cell proliferation through c-Myc signaling [12]. Barroilhet *et al*. found that CtBP2 was aberrantly elevated in human ovarian tumors and that CtBP2 expression accelerated tumor cell growth and mobility [13]. Similar findings have also been reported in breast cancer studies that examined CtBP2 expression [14, 15]. However, the mechanism governing CtBP2 overexpression in cancer remains unclear.

Glioma-associated oncogene 1 (GLI1) is a downstream transcription factor in the hedgehog signaling pathway that reportedly accelerates the progression of various cancers, including basal cell carcinoma [16], colon cancer [17], medulloblastoma [18], gastric cancer [19] and pancreatic carcinoma [20]. We previously reported GLI1 overexpression in HCC tissues and were able to predict rapid tumor recurrence after surgery using GLI1 expression levels. GLI1 consists of a conserved C2H2 zinc finger DNA-binding domain that specifically interacts with a GACCACCCA-like motif in the promoters of various target genes. GLI1 mediates the expression of a variety of important cancer progression genes, including SNAI1 [21], ABCG2 [22], CYLD, DNMT [23], RegIV [24], AKT [25] and Caveolin-1 [26]. We demonstrated that aberrantly upregulated GLI1 promoted HCC progression by regulating epithelial-mesenchymal transition (EMT) through the GLI1 transcriptional target Snail Family Zinc Finger 1 (SNAI1) [21]. We found seven potential GLI1 binding sites in the CtBP2 promoter, which lead us to hypothesize that GLI1 overexpression might contribute to the upregulation of CtBP2 in HCC.

We report that CtBP2 expression was upregulated in the HCC tissues examined in this study, and that elevated CtBP2 expression was associated with elevated GLI1 expression and poor overall postsurgical survival. We verified that CtBP2 was directly upregulated by GLI1 *in vitro*, and demonstrated that the upregulated CtBP2 bound the PQDLSLK motif of SNAI1 in the nucleus. Additionally, the oncogenic Role of CtBP2 was validated using a HCC xenograft model. Therefore, the findings of this study indicate that CtBP2 might facilitate GLI1-SNAI1 induced EMT in HCC. This is the first report describing the mechanism underlying CtBP2 overexpression, identifying the role played by CtBP2 in EMT in HCC and showing CtBP2 is an effective predictive biomarker of patient outcome after HCC surgery.

## RESULTS

### CtBP2 was overexpressed in HCC and overexpression predicted poor post-surgical outcomes

We examined tumor tissues and adjacent liver tissues from 100 HCC patients for CtBP2 expression by immunohistochemistry. We found that CtBP2 staining was strongest in the tumor cell cytoplasm, while nuclear staining was observed in relatively few cells (Figure 1A). CtBP2 expression was elevated in tumor cells when compared to benign tissues in 60% of the HCC tumors examined. Mann-Whitney U analysis demonstrated that CtBP2 expression was significantly higher in HCC tissues when compared to adjacent liver tissues (*p* < 0.001, Figure 1B). Clinical association analysis using the Spearman rank test demonstrated that CtBP2 overexpression in HCC tissues was positively correlated with tumor size ( *p* = 0.039), venous infiltration ( *p* = 0.003), Edmondson-Steiner Classification ( *p* < 0.001) and the Tumor Node Metastasis (TNM) stage (* p* = 0.018).

**Figure 1:** CtBP2 expression was upregulated in HCC tissues and associated with poor prognosis after liver resection **(A)** CtBP2 was expressed mainly in the cytoplasm of tumor cells and CtBP2 expression was notably higher in HCC tissues (a) when compared to matched normal adjacent liver tissues (b). **(B)** The Mann–Whitney *U* test confirmed that CtBP2 expression was significantly higher in HCC tissues than adjacent liver tissues from 100 HCC patients (* p* < 0.001). **(C)** Kaplan Meier overall survival curves indicated that the High CtBP2 Group had an obviously shortened post-surgical survival time when compared to the Low CtBP2 Group (HR = 3.071; 95% CI: 1.357, 6.951; *p* = 0.007). **(D)** There was more GLI1 expression in HCC tissues (a) compared to matched normal adjacent liver tissues (b), and most of the GLI1-positive cells showed nuclear staining. **(E)** SNAI1 expression was notably increased in HCC tissues by IHC (a) when compared to matched adjacent healthy liver tissues (b). **(F)** The Spearman rank test indicated that GLI1 expression correlated positively with CtBP2 expression (*r* = 0.701, *p* < 0.001, left panel) and SNAI1 (*r* = 0.759, *p* < 0.001, right panel) in HCC tissues, respectively.

Post-surgical follow-up information was collected from 87 of the original 100 HCC patients and Kaplan–Meier survival curves were constructed. The median overall survival was 14.8 months for HCC patients with elevated tumor tissue CtBP2 expression (High CtBP2 Group), whereas the median overall survival was 58.3 months for HCC patients with lower CtBP2 levels in adjacent liver tissues (Low CtBP2 Group). The three-year survival rate was 30.9% in the High CtBP2 Group compared to 70.7% in the Low CtBP2 Group. Similarly, patients in the High CtBP2 Group (23.6%) had a reduced five-year survival rate when compared to patients from the Low CtBP2 Group (41.9%). Overall survival curve comparisons indicated that the High CtBP2 Group patients had a significantly worse prognosis when compared to patients from the Low CtBP2 Group (HR = 3.071; 95% CI: 1.357, 6.951; *p* = 0.007; Figure 1C). Univariate analysis demonstrated that venous infiltration, higher Edmondson-Steiner classification, advanced TNM staging and higher CtBP2 expression in tumor tissues were the poor prognosis factors (Table 2). Moreover, multivariate Cox proportional-hazard regression analysis indicated that venous infiltration, advanced TNM staging and higher CtBP2 expression in tumor tissues were independent prognostic factors (Table 2). These data indicated that CtBP2 overexpression in HCC tissues was a predictor of poor survival outlook after liver resection. To investigate whether there was a correlation between CtBP2 and GLI1 protein expression in HCC tissues, we conducted immunohistochemical (IHC) analysis of GLI1 expression in the clinical samples. As shown in Figure 1D, GLI1 was upregulated in HCC tissues when compared to adjacent liver tissues, which was consistent with the results of previous investigations [21, 26]. Similarly, SNAI1 expression was significantly elevated in HCC tissues when compared to adjacent liver tissues (Figure 1E). Spearman rank analysis positively associated elevated GLI1 expression with CtBP2 and SNAI1 in HCC tissues (*r* = 0.701, *p* < 0.001, Figure 1F). This result raised the possibility that GLI1 expression could be related to the overexpression of both CtBP2 and SNAI1 in HCC.

### CtBP2 expression in HCC cell lines

To examine CtBP2 expression in HCC cell lines and to identify the most appropriate HCC cell model for further investigations, we conducted qRT-PCR assays and Western blots to detect CtBP2 mRNA and protein expression, respectively, in Hep3B, PLC/PRF/5, HepG2, MHCC97H and Huh7 cells. All five HCC cell lines expressed different CtBP2 levels (Figure 2A). When compared to the Huh7 and Hep3B cell lines, CtBP2 mRNA expression was higher in MHCC97H, PLC/PRF/5 and HepG2 cells. CtBP2 protein expression, as measured by Western blotting, mirrored the mRNA expression in all five HCC cell lines (Figure 2B). The Huh7 and MHCC97H cell lines had the lowest and the highest CtBP2 expression levels, respectively. Therefore, we selected the Huh7 cell line for the CtBP2 overexpression experiments in this study, and the MHCC97H cell line was used for the CtBP2 knockdown experiments.

**Figure 2:** The expression of CtBP2 in HCC cell lines **(A)** CtBP2 mRNA levels in five different HCC cell lines was assessed by qRT-PCR. **(B)** CtBP2 protein expression in five different HCC cell lines was examined by Western blotting.

### CtBP2 promoted HCC cell migration and invasion by inducing EMT

To investigate the mechanism underlying CtBP2 promotion of HCC progression, we increased CtBP2 expression in Huh7 cells by stably transfecting the Huh7 cell line with a CtBP2 expressing plasmid. Successful transfection was confirmed by both qRT-PCR and Western blotting (Figure 3A). Wound healing assays demonstrated that the migration rate of Huh7 cells stably transfected with the CtBP2 expressing plasmid (Huh7 CtBP2 cells) was notably faster than Huh7 cells transfected with a vector plasmid control (Huh7 Vector cells) 24 and 48 h after scratching the cell layer (Figure 3B). To assess invasiveness, we conducted Transwell invasion assays and observed that Huh7 cell invasiveness was significantly increased by increased CtBP2 expression (Figure 3C).

**Figure 3:** Elevated CtBP2 expression promoted Huh7 cell mobility and invasion by inducing EMT **(A)** Both qRT-PCR and Western blotting assays verified that CtBP2 expression was increased after stable transfection of CtBP2 expression plasmid. **(B)** The migration capacity of Huh7 cells, as assessed by wound healing assays, was enhanced by CtBP2 overexpression. **(C)** Transwell invasion assays demonstrated that elevating CtBP2 expression increased the invasive capability of Huh7 cells. **(D)** Overexpression of CtBP2 decreased E-cadherin expression and increased the expression of N-cadherin, Vimentin and Fibronectin in Huh7 cells, as measured by Western blotting. **(E)** Double immunofluorescence staining confirmed that CtBP2 overexpression resulted in the downregulation of E-cadherin and the upregulation of N-cadherin in Huh7 cells.

To investigate whether CtBP2 expression accelerated HCC cell mobility and invasiveness by inducing EMT, we examined the expression of EMT biomarkers in Huh7 cells using Western blotting and immunofluorescence staining. The biochemical markers examined included E-cadherin (which is expressed predominantly in epithelial cells), and N-cadherin, Vimentin and Fibronectin (which are expressed predominantly in mesenchymal cells). The Western blotting indicated that elevated CtBP2 expression attenuated E-cadherin expression, but increased N-cadherin, Vimentin and Fibronectin expression in Huh7 cells (Figure 3D). We performed double immunofluorescence staining to confirm the Western blotting experiments and observed reduced E-cadherin and elevated N-cadherin expression in Huh7 CtBP2 cells compared to the control Huh7 Vector cells (Figure 3E).

To verify the role of CtBP2 on EMT in HCC, we used CtBP2 targeted siRNAs to silence CtBP2 expression in MHCC97H cells (Figure 4A). Consistent with the results in the Huh7 cell experiments, CtBP2 knockdown suppressed the migration and invasion of MHCC97H cells (Figure 4B and 4C). Additionally, we observed that CtBP2 suppression lead to E-cadherin upregulation in MHCC97 cells, but decreased the expression of N-cadherin, Vimentin and Fibronectin (Figure 4D). Taken together, these data strongly support the hypothesis that CtBP2 promotes HCC cell mobility and invasion by inducing EMT.

**Figure 4:** CtBP2 knockdown inhibited MHCC97H cell migration and invasion capacities by repressing EMT **(A)** Both qRT-PCR and Western blotting assays confirmed that siRNA transfection eliminated CtBP2 expression in MHCC97H cells. **(B)** Wound healing assays indicated that CtBP2 siRNA suppressed MHCC97H cell migration. **(C)** The invasive ability of MHCC97H cells was repressed by CtBP2 siRNA in Transwell invasion assays. **(D)** Western blotting assays demonstrated that CtBP2 suppression lead to E-cadherin upregulation and N-cadherin, Vimentin and Fibronectin downregulation in MHCC97H cells.

### GLI1 upregulated CtBP2 transcription by binding with its promoter

Our preliminary investigations suggested that GLI1 plays a critical role in the EMT phenotype of HCC cells and the results of the current study strongly indicated that CtBP2 might be involved in EMT in HCC. Therefore, we next investigated whether the transcription factor GLI1 regulates CtBP2 expression. We stably transfected Huh7 cells with a GLI1 expressing vector or an empty control vector and observed that elevated GLI1 expression significantly enhanced CtBP2 expression (Figure 5A). Next, using MatInspector professional version 7.2, we identified several potential GLI binding sites in the CtBP2 promoter (Figure 5B). To determine whether GLI1 could directly interact with the CtBP2 promoter and to identify the core promoter region of CtBP2, we cloned four CtBP2 promoter fragments (pGL3−2000, −2000/−1 bp; pGL3−1307, −1307/−1 bp; pGL3−675, −675/−1 bp; pGL3−1350, −1350/−652 bp) into a luciferase reporter vector and conducted a luciferase reporter assay in Huh7 cells stably transfected with the GLI1 expressing plasmid. The four reporter plasmids each displayed different levels of promoter activity, but all displayed notably stronger promoter activity than the pGL3-basic control plasmid (Figure 5C). The pGL3−1307 plasmid displayed the strongest promoter activity. Remarkably, when the fragment between −1307 bp and −676 bp was deleted, the luciferase activity was almost abolished. The pGL3−1350 plasmid containing the −1350/−652 bp CtBP2 promoter fragment displayed the second highest promoter activity level of the transfected Huh7 CtBP2 cells. These data suggested the existence of a critical positive regulatory element in the −1350/−652 bp CtBP2 promoter fragment. To further investigate the importance of the −1350/−652 bp CtBP2 promoter fragment we examined pGL3−1350 luciferase activity in Huh7 cells transfected with a GLI1 expressing plasmid (Huh7 GLI1) or a control plasmid (Huh7 Vector). We observed that elevated GLI1 expression increased the luciferase activity of the pGL3−1350 reporter plasmid (Figure 5D).

**Figure 5:** GLI1 increased CtBP2 expression directly by binding to its promoter **(A)** Both qRT-PCR and Western blotting assays demonstrated that the expression of GLI1 (left panel) and CtBP2 (right panel) were notably elevated after GLI1 overexpression in Huh7 cells. **(B)** A schematic model of the locations and sequences of the 14 potential GLI1 binding sites (BS). The consensus GLI1 binding sequence is listed here. **(C)** Luciferase reporter assays in Huh7 GLI1 cells indicate that the pGL3−1307 (−1307/−1 bp CtBP2 promoter fragment) has the strongest promoter activity. When the fragment between −1307 bp and −676 bp was deleted, the luciferase activity greatly reduced. The pGL3−1350 (−1350/−652 bp CtBP2 promoter fragment) displayed the second highest level of promoter activity. **(D)** Luciferase reporter assays demonstrated that the luciferase activity of pGL3−1350 was notably enhanced after GLI1 overexpression in Huh7 cells. This supports the ability of the GLI1 protein to bind the CtBP2 promoter in the −1350/−652 bp region. **(E)** DNA fragments capable of binding the GLI1 protein in the cell nucleus were analyzed by ChIP assay. As the upper panel shows, the PCR assay showed that the GLI1 protein was capable of directly binding to the −1350/−652 bp CtBP2 promoter fragment. After equalization using RNA Polymerase II (Input), more CtBP2 promoter fragment was bound to the GLI1 protein in Huh7 GLI1 cells. Similarly, a relative rtPCR assay demonstrated that elevated GLI1 expression increased the CtBP2 promoter occupancy of GLI1 in Huh7 cells, as presented in the lower panel.

A ChIP assay further supported the hypothesis that the GLI1 protein directly interacted with and bound the −1350/−652 bp CtBP2 promoter fragment. Overexpression of GLI1 increased the CtBP2 promoter occupancy of GLI1 in Huh7 cells (Figure 5E). Therefore, the results of our experiments implied that GLI1 mediates CtBP2 expression by directly binding its promoter in HCC cells.

### CtBP2 acted as a transcriptional co-repressor and its recruitment was critical for GLI1/SNAI1 induction of the HCC EMT phenotype

To investigate whether CtBP2 directly induced EMT, we examined the relationship between CtBP2, SNAI1 and EMT in HCC. We abolished SNAI1 expression in Huh7 cells using SNAI1 siRNA [21] and induced CtBP2 expression with transfection of a CtBP2 expressing plasmid (Figure 6A). In the absence of SNAI1, CtBP2 overexpression did not affect the expression of E-cadherin, N-cadherin, Vimentin or Fibronectin as much as it did in cells expressing normal levels of SNAI1, as presented in Figure 6B. This result indicated that SNAI1 was required for CtBP2-driven EMT and that CtBP2 was not a direct mediator of EMT in HCC.

**Figure 6:** CtBP2 interacted with SNAI1 and played a critical role in GLI1/SNAI1 induction of EMT **(A)** Both qRT-PCR and Western blotting assays demonstrated that SNAI1 siRNA abated SNAI1 expression (left panel) in Huh7 cells and that CtBP2 expression was enhanced by CtBP2 expression plasmid transfection in Huh7 cells without SNAI1. **(B)** Western blotting showed that CtBP2 overexpression lead to E-cadherin downregulation and N-cadherin, Vimentin and Fibronectin upregulation in Huh7 cells with normal SNAI1 expression. However, silencing SNAI1 counteracted the regulatory effect of CtBP2 on E-cadherin, N-cadherin, Vimentin and Fibronectin. **(C)** Co-IP assays demonstrated direct CtBP2 and SNAI1 binding in Huh7 GLI1 cells. **(D)** Both qRT-PCR and Western blotting verified that siRNA abolished CtBP2 expression in Huh7 GLI1 cells. **(E)** Western blotting assays demonstrated that CtBP2 knockdown in Huh7 GLI1 cells lead to E-cadherin upregulation and N-cadherin, Vimentin and Fibronectin downregulation, while SNAI1 expression was not significantly affected. However, silencing CtBP2 did not affect the expression of E-cadherin, N-cadherin and Fibronectin. Neither the expression of Vimentin nor the expression of SNAI1 could be detected in Huh7 Vector cells transfected with CtBP2 siRNAs or Scr siRNAs.

Recent studies have reported that CtBP2 is recruited to the E-cadherin promoter and modulates its transcription [29]. The Levine group demonstrated that the CtBP2 interaction motif P-DLS-K is present in the repression domains of SNAI1 [30]. Due to the increased SNAI1 expression we found in our previous study [21] and the enhanced CtBP2 expression observed in Huh7 GLI1 cells in this study, we conducted a Co-IP assay to observe whether CtBP2 and SNAI1 directly interact. We found that the CtBP2 protein bound the SNAI1 protein in the nucleus of Huh7 GLI1 cells (Figure 6C). To investigate the role of CtBP2 in GLI1/SNAI1 driven EMT, we used expression in Huh7 GLI1 cells (Figure 6D). We found that E-cadherin expression was increased in the siRNA CtBP2 silenced cells, that the expression of N-cadherin, Vimentin and Fibronectin were repressed, and that SNAI1 expression was not significantly altered (Figure 6E). On the other hand, CtBP2 knockdown in Huh7 Vector cells did not affect the expression of aforementioned EMT markers clearly. These data indicated that CtBP2 bound SNAI1 as a transcriptional co-repressor and, thereby, promoted GLI1/SNAI1 driven EMT in HCC.

### CtBP2 accelerated tumor growth and promoted EMT in the HCC xenograft model

To further study the role of CtBP2 in HCC progression, we conducted HCC xenograft experiments in nude mice. Huh7 CtBP2 and Huh7 Vector cells were subcutaneously injected into six nude mice. The growth of xenograft tumors was observed weekly using calipers and tumors were harvested after four weeks. The xenograft tumors derived from the Huh7 CtBP2 cells (Huh7 CtBP2 Group) were notably larger than those derived from the Huh7 Vector cells (Huh7 Vector Group) (Figure 7A). Unpaired Student's *t*-tests confirmed that the xenograft tumors obtained from the Huh7 CtBP2 Group were remarkably larger than the tumors obtained from the Huh7 Vector Group ( *p* = 0.001, Figure 7B). IHC staining demonstrated significantly stronger N-cadherin expression and less E-cadherin expression in the Huh7 CtBP2 Group's xenograft tumors (Figure 8). We did not observe upregulation of either GLI1 or SNAI1 in the Huh7 CtBP2 Group, providing evidence that CtBP2 did not mediate either GLI1 or SNAI1 expression in xenograft HCC tumors. In summary, these results supported the hypothesis that CtBP2 promotes tumor progression and induces the EMT phenotype in HCC.

**Figure 7:** Elevated CtBP2 expression accelerated HCC xenograft growth and promoted EMT in HCC xenograft tissues **(A)** Representative pictures of HCC xenografts from both Huh7 Vector (left panel) and Huh7 CtBP2 cells (right panel). **(B)** Xenograft size in the Huh7 CtBP2 group was significantly larger than in the Huh7 Vector Group ( *p* = 0.001).

**Figure 8:** Compared to the Huh7 Vector group, there was more CtBP2 and N-cadherin protein expression in xenograft tissues from the Huh7 CtBP2 group, whereas E-cadherin expression was decreased GLI1 and SNAI1 expression was undetected in xenograft tissues from either the Huh7 CtBP2 or the Huh7 Vector Group.

## DISCUSSION

We have identified a role for CtBP2 in the progression of HCC and revealed a correlation between CtBP2 expression in HCC tissues and patient prognosis after liver resection. We report six novel discoveries in this study: (1) CtBP2 was upregulated in HCC tissues when compared to matched adjacent healthy liver tissues and CtBP2 overexpression in HCC tissues was correlated with poor patient prognosis; (2) CtBP2 overexpression promoted cell motility and invasion by inducing EMT in HCC cells; (3) GLI1 bound the CtBP2 promoter directly and increased its expression, which is potentially the underlying mechanism of CtBP2 upregulation in HCC; (4) CtBP2 bound SNAI1, a well-known EMT inducer, and was required as a transcriptional co-repressor for GLI1/SNAI1 driven EMT in HCC cells; (5) SNAI1 was also essential for CtBP2 induced EMT in HCC cells; (6) CtBP2 overexpression accelerated tumor growth and promoted EMT in HCC xenograft tumors. In summary, the results of this study strongly support the potential of CtBP2 as a predictive factor of patient outcome after liver resection and as a therapeutic target for the treatment of HCC.

EMT is a fundamental cellular process that is involved in epithelial tissue morphogenesis during tissue development and cancer progression. In our previous studies, we demonstrated that EMT was critical to HCC progression and regulated by the GLI1/SNAI1 axis [21, 26, 27]. To reveal the mechanism through which GLI1 and SNAI1 mediate EMT in HCC, we investigated the role of CtBP2 in GLI1/SNAI1 axis induced EMT.

CtBP2 was initially discovered as a phosphoprotein bound to the C-terminal of the adenovirus E1A protein. It was recently reported to function as a transcriptional co-repressor that binds various transcriptional repressors with PXDLS binding motifs. In turn, these transcriptional repressors target and suppress the expression of multiple tumor repressors, including E-cadherin [31], PTEN [32] and p16Ink4a [33]. Using both *in vitro* and *in vivo* experiments, we demonstrated that CtBP2 overexpression induced EMT in HCC and promoted cell migration and invasion. After searching the RCSB Protein Data Bank, we found that the SNAI1 protein contained the PQDLSLK motif. The presence of this motif implied that the CtBP2 protein was potentially a binding partner of the SNAI1 protein and that CtBP2 might function as a transcriptional co-repressor. The Co-IP results confirmed this hypothesis. Additionally, the *in vitro* experiments revealed that CtBP2 knockdown reversed GLI1/SNAI1 driven EMT, but CtBP2 could not induce EMT in HCC cells without SNAI1 expression. Interestingly, we found that enhanced GLI1 expression promoted CtBP2 upregulation. Fourteen potential GLI1-binding sites were observed in the CtBP2 promoter after searching the RCSB Protein Data Bank. ChIP and luciferase reporter assays suggested that GLI1 bound the −1350/−652 bp CtBP2 promoter fragment. These data indicated that GLI1 directly promoted CtBP2 expression. Therefore, we concluded that SNAI1 and CtBP2 both promoted the EMT phenotype of HCC cells, could directly interact with one another and were both directly upregulated by GLI1.

This investigation also reported aberrant over-expression of CtBP2 in HCC tissues when compared to matched normal adjacent liver tissues. After analyzing the patient follow-up data, we determined that CtBP2 overexpression in HCC tissues predicted poor patient prognosis after liver resection. The highly significant results of this analysis suggest that CtBP2 could be a useful prognostic marker of patient outcome after HCC surgery. Our clinical investigation also revealed that there was positive association between GLI1 and CtBP2 expression in HCC tissues, further supporting our conclusion that GLI1 upregulates CtBP2 expression in HCC.

In summary, as illustrated in Figure 9, we have identified a novel function for CtBP2 as a transcription co-repressor that interacts with SNAI1 and contributes to inducing the EMT phenotype of HCC cells. We found that GLI1 upregulated both SNAI1 and CtBP2. This upregulation results in the induction of EMT, and, therefore, this study characterizes the mechanism by which GLI1 modulates the EMT in HCC. Finally, CtBP2 appears to be an effective predictive factor for HCC outcome after liver resection and additional future studies developing CtBP2 as a prognostic marker, in addition to studies investigating its potential as an HCC treatment target, should be conducted.

**Figure 9:** Working model of the role of CtBP2 in EMT induced by the GLI1/SNAI1 axis in HCC GLI1 upregulates both SNAI1 and CtBP2 simultaneously. SNAI1 binds the E-cadherin promoter after binding CtBP2, leading to the EMT phenotype of HCC cells.

## METHODS

### Clinical samples

One hundred patients diagnosed with HCC between January 2004 and June 2006 in the Department of Hepatobiliary Surgery at the First Affiliated Hospital of Xi'an Jiaotong University were recruited in this investigation. Written informed consent was obtained from all patients and all protocols in this study were approved by the Xi'an Jiaotong University Ethics Committee according to the Helsinki Declaration of 1975. None of the patients enrolled in this study had undergone pre-operative chemotherapy or embolization. After routine diagnostic procedures, including X-ray, abdominal ultrasonography and computed tomography, all patients received surgical treatment, including curative resection for early HCC and palliative resection for advanced HCC. HCC samples and paired adjacent liver samples (> 2 cm distance from the margin of the resected tissue) were obtained during each liver resection and immediately fixed in paraformaldehyde for immunohistochemistry. Clinical data from these 100 HCC patients were collected from their medical records. An experienced pathologist performed the HCC diagnosis, Edmondson classification, clinical tumor-node-metastasis (TNM) grading and measured maximum tumor diameter. After surgery, all patients were followed for 15 to 120 months. Follow-up information was successfully obtained from 87 patients. The demographic features and clinicopathological data are presented in Table 1.

**Table 1:** Correlation between clinicopathological characteristics and CtBP2 overexpression in the tumor tissues of 100 HCC patients

Clinicopathological features		No. of patients		χ^2^	*p*
		Higher CtBP2	Lower CtBP2		
Age (year)	< 50	20	12	0.12	0.726
	≧ 50	40	28		
Gender	Male	48	30	0.35	0.554
	Female	12	10		
HBV infection	Present	50	32	0.18	0.671
	Absent	10	8		
Serum AFP level (ng/mL)	≧ 400	46	27	1.02	0.312
	< 400	14	13		
Tumor size (cm)	≧ 5	51	27	4.28	0.039
	< 5	9	13		
Liver cirrhosis	Present	56	33	2.88	0.089
	Absent	4	7		
Venous infiltration	Present	30	8	9.17	0.003
	Absent	30	32		
Edmondson-Steiner Classification	I + II	6	21	21.99	< 0.001
	III + IV	54	19		
TNM stage	I + II	38	34	5.59	0.018
	III + IV	22	6		

**Table 2:** Cox regression analysis of the correlation between clinicopathological features and the overall postsurgical survival rate of HCC patients

Clinicopathological features	Unvariate Analysis		Multivariate Analysis	
	RR (95% CI)	*p* Value	RR (95% CI)	*p* Value
Venous infiltration	4.320 (2.043 – 6.875)	0.018	3.562 (1.750 – 4.895)	0.025
Higher Edmondson-Steiner classification	2.322 (1.252 – 3.210)	0.003	1.854 (0.899 – 2.152)	0.010
Advanced TNM staging	3.232 (2.012 – 4.365)	0.008	1.989 (1.228 – 3.788)	0.030
Higher CtBP2 in tumor tissue	3.689 (1.922 – 5.025)	0.021	3.025 (1.752 – 6.982)	0.001

### Cell lines

The Hep3B, PLC/PRF/5 and HepG2 human HCC cell lines were obtained from the Institute of Biochemistry and Cell Biology at the Chinese Academy of Sciences (Shanghai, China). The MHCC97H cells were obtained from Fudan University (Shanghai, China). The Huh7 cells were a kind gift from Prof. Kefeng Dou (Department of Hepatobiliary Surgery, Xijing Hospital, Fourth Military Medical University). Hep3B and PLC/PRF5 cells were cultured in complete MEM medium with 10% fetal bovine serum (FBS). MHCC97H and Huh7 cells were grown in DMEM with 10% FBS. HepG2 cells were cultured in RPMI 1640 medium with 10% FBS. All HCC cells were grown in a humidified incubator with 5% CO2 at 37°C.

### Expression vectors

CtBP2 expressing plasmids and GLI1 expressing plasmids were generated by cloning the respective cDNA into pCMV-Tag2B vectors purchased from Stratagene (Santa Clara, CA, USA). The sequence of both expression plasmids were confirmed by polymerase chain reaction (PCR) and Western blotting.

### Western blotting

Protein expression was examined by Western blotting. Cell lysates (50 μg) were prepared in RIPA buffer…The following antibodies were used: mouse monoclonal antibodies to E-cadherin (Santa Cruz, CA, USA), Vimentin (Santa Cruz), β-actin (Boster Biotechnology, Wuhan, China) and rabbit polyclonal antibodies against GLI1, SNAI1, N-cadherin and CtBP2 (Abcam, Cambridge, UK).

### Quantitative real-time reverse transcription polymerase chain reaction (qRT-PCR)

HCC cells were cultured to 80% confluence, washed with ice-cold PBS and subjected to RNA extraction using 1 ml of Trizol (Invitrogen, NY, USA). cDNA synthesis was carried out with the High Capacity cDNA Reverse Transcription Kit from Applied Biosystems (Carlsbad, CA, USA) and ABI TaqMan Gene Expression assays were carried out for qRT-PCR using the 7300 Real-Time PCR System (Applied Biosystems). 18S ribosomal RNA (rRNA) was measured as an internal control and the mRNA levels of target genes were normalized to the 18S rRNA level in the same sample.

### Immunofluorescence and confocal microscopy

HCC cells were plated on cover slips overnight, fixed for 20 min with 2.5% formaldehyde in PIPES buffer and then treated with 0.25% Triton X-100 for 15 min. After incubating the slides in blocking buffer (5% normal goat serum and 5% glycerol in D-PBS) for 1 h at 37°C, they were incubated with mouse anti-E-cadherin and rabbit anti-N-cadherin antibodies at 4°C overnight followed by washing with PBS three times. Cover slips were then incubated with Alexa-Fluor-555 conjugated donkey anti-rabbit and Alexa-Fluor-488 conjugated goat anti-mouse secondary antibodies at room temperature for 60 min, followed by DAPI nuclear counterstaining for 10 min. Images were taken by confocal microscopy (Carl Zeiss, Oberkochen, Germany).

### Migration assay

Cell mobility was determined with a wound healing assay. As described previously [27], HCC cells were grown to full confluence in 24-well plates. After the cells had grown to confluency a “wound” was created by scratching the length of the well with a 1,000 μl pipette tip. Images were captured with an inverted digital camera at 0, 24 and 48 h. Cell migration was quantitated by measuring the width of the wound at each time point. Each assay was replicated three times.

### Transwell invasion assay

Matrigel was diluted 1:3 in serum-free medium before being added to the upper chamber of a 24-well Transwell plate (Millipore, Billerica, Massachusetts, USA). HCC cells were trypsinized and counted manually under a microscope. A cell suspension of 50,000 cells/mL in serum-free medium was prepared and 100 μL of the suspension was loaded into the top chamber. The bottom chambers were filled with medium with 10% FBS. Invasion was halted after 24 hrs incubation in a 37°C incubator (5% CO2) by scraping the non-migrated cells off the upper chamber using a cotton swab. After being fixed in 4% paraformaldehyde, migrated cells were stained with 0.05% Crystal Violet. Migrated HCC cells were counted under an inverted light microscope.

### Chromatin immunoprecipitation assay (ChIP assay)

HCC cells were cross-linked with 1% formaldehyde for 10 min at room temperature before the ChIP assay. The EZ-Magna ChIPTM Chromatin Immunoprecipitation Kit was purchased from Millipore for the ChIP assay. According to the manufacturer's instructions, proteins were cross-linked with 1% formaldehyde after cell lysis and DNA shearing with 15 cycles of sonication. Next, immunoprecipitation was conducted using the GLI1 antibody (Cell Signaling Technology, Danvers, MA, USA), normal rabbit IgG (Santa Cruz) as a negative control (IgG group) and anti-RNA Polymerase II antibody as the positive control (Input group). Following immunoprecipitation, cross-links were removed and immunoprecipitated DNA was purified and then amplified by qRT-PCR using the SYBR Green PCR Master Mix (Applied Biosystems). The primers used to detect the CtBP2 promoter were designed as follows: Forward: 5′-GCCGAACTCAGGGTAGTGAG-3′; Reverse: 5′-CGT CCTGACGTCTCAAGGTT-3′.

### Luciferase reporter assay

Four CtBP2 promoter fragments (−2000/−1 bp, −1307/−1 bp, −675/−1 bp and −1350/−652 bp from the transcription start site) were isolated by PCR amplification and ligated into the luciferase reporter vector pGL3-Basic from Promega (Fitchburg, WI, USA). Huh7 cells were plated on 24-well plates one day prior to the transfection. Huh7 cells were co-transfected with luciferase promoter reporter vectors and GLI1 expressing plasmids. After 48 hours, luciferase activity was examined using the Dual-Luciferase Reporter Assay System (Promega) according to the manufacturer's protocol.

### Co-immunoprecipitation assay (Co-IP assay)

The co-immunoprecipitation assay was performed using Huh7 cells transfected with GLI1 expressing plasmid (Huh7 GLI1 cells). Protein lysate was extracted in immunoprecipitation buffer (50 mM Tris–HCl, pH 8.0, 150 mM NaCl, 5 mM EDTA, 0.5% NP-40, 2 μg/ml aprotinin, 1 μg/ml leupeptin, 1 mM PMSF, 1 mM sodium vanadate and 10 mM sodium fluoride). For Co-IP, 10 μl protein A/G-agarose beads pre-conjugated with the antibody against CtBP2 or SNAI1 and IgG were utilized to isolate the immunocomplexes. The antibody-conjugated beads were shaken with cell lysates at 4°C overnight. The next day, isolated beads were washed twice with PBS buffer and twice with RIPA buffer. The supernatant was examined by Western blotting.

### Immunohistochemical (IHC) staining

IHC staining was conducted as described previously [28]. Paraffin embeded samples were cut into 4 μm-thick sections, which were then deparaffinized in xylene and re-hydrated. The slices were incubated in 0.3% hydrogen peroxide for 30 min to block endogenous peroxidase activity and then antigen retrieval was performed in sodium citrate buffer for 45 s in a pressure cooker. After overnight blocking at 4°C, sections were incubated with primary antibodies against CtBP2 or GLI1 at 4°C overnight. Bound primary antibodies were detected using biotinylated secondary antibodies (Zhongshan Goldenbridge Biotechnology Lltd. Co., Beijing, China). Next, sections were incubated with diaminobenzidine before being counterstained with hematoxylin. Finally, sections were dehydrated in alcohol and xylene.

Sections were independently evaluated by two experienced pathologists. Staining intensity was scored using four grades (0 – 3): 0 (negative), 1 (weakly positive), 2 (moderately positive) and 3 (strongly positive). The percentage of positive cells was also scored using five categories (0 – 4): a score of 0 was given for 0 – 5%, 1 for 6 – 25%, 2 for 26 – 50%, 3 for 51 – 75%, and 4 for > 75%. The final staining score was obtained by multiplying the staining intensity and the percentage of positive cells.

### *In vivo* tumorigenesis assay

5 × 10^6^ Huh7 cells were transfected using control or CtBP2 expressing plasmids before being subcutaneously injected into the flanks of 4-week-old male BALB/c nude mice (Centre of Laboratory Animals, The Medical College of Xi'an Jiaotong University, Xi'an, China). Tumor sizes were measured weekly using calipers and calculated with the following formula: volume = A × B^2^ × 0.52 (A, length; B, width; all measurements were in millimeters). After four weeks, the mice were sacrificed by cervical dislocation under anesthesia. All *in vivo* experimental protocols were approved by the institutional animal care and use committee of the First Affiliated Hospital of Xi'an Jiaotong University.

### Statistical analysis

CtBP2 protein expression levels in HCC tissues and matched normal adjacent liver tissues were compared using the Mann-Whitney *U* test. The correlation between CtBP2 and GLI1 expression levels was analyzed using Spearman rank test. The Kaplan–Meier curves of HCC patients were assessed using the log-rank test. A *p* value of < 0.05 was considered significant. Multivariate analysis was performed using SPSS Version 17.0 software (SPSS Inc., Chicago, IL, USA). PRISM 5 software (GraphPad, La Jolla, CA, USA) was used for all other statistical analyses.

## Abbreviations

CtBP: C-terminal binding protein
HCC: hepatocellular carcinoma
GLI1: GLI family zinc finger 1
EMT: epithelial-mesenchymal transition
PBS: Phosphate buffered saline
FBS: Fetal bovine serum
Co-IP: Co-immunoprecipitation
ChIP: Chromatin Immunoprecipitation
IHC: Immunohistochemistry
